# A Joint Model for Unbalanced Nested Repeated Measures with Informative Drop-Out Applied to Ambulatory Blood Pressure Monitoring Data

**DOI:** 10.1155/2022/4452158

**Published:** 2022-02-25

**Authors:** Enas M. Ghulam, Jane C. Khoury, Roman Jandarov, Raouf S. Amin, Eleni-Rosalina Andrinopoulou, Rhonda D. Szczesniak

**Affiliations:** ^1^Basic Science Department, College of Science and Health Professions, King Saud bin Abdulaziz University for Health Sciences, Jeddah, Saudi Arabia; ^2^King Abdullah International Medical Research Center, Jeddah, Saudi Arabia; ^3^Division of Biostatistics and Epidemiology, Cincinnati Children's Hospital Medical Center, Cincinnati, USA; ^4^Department of Environmental Health, University of Cincinnati, Cincinnati, USA; ^5^Department of Pediatrics, Cincinnati Children's Hospital Medical Center, Cincinnati, USA; ^6^Division of Pulmonary Medicine, Cincinnati Children's Hospital Medical Center, Cincinnati, USA; ^7^Department of Biostatistics, Department of Epidemiology, Erasmus Medical Center, Rotterdam, Netherlands

## Abstract

This study proposes a Bayesian joint model with extended random effects structure that incorporates nested repeated measures and provides simultaneous inference on treatment effects over time and drop-out patterns. The proposed model includes flexible splines to characterize the circadian variation inherent in blood pressure sequences, and we assess the effectiveness of an intervention to resolve pediatric obstructive sleep apnea. We demonstrate that the proposed model and its conventional two-stage counterpart provide similar estimates of nighttime blood pressure but estimates on the mean evolution of daytime blood pressure are discrepant. Our simulation studies tailored to the motivating data suggest reasonable estimation and coverage probabilities for both fixed and random effects. Computational challenges of model implementation are discussed.

## 1. Introduction

Hypertension is one of the major causes and most important modifiable risk factors for the prevention of cardiovascular disease. Hypertension affects an estimated 1 billion people worldwide [1]. Ambulatory blood pressure monitoring (ABPM) is a critical measurement technique to monitor blood pressure in the home environment by obtaining multiple readings over a 24-hour period [1, 2]. Sequences of ABPM measurements are often recorded intensively over a period of time, under different medical conditions or occasions on the same subject to assess the variation of these sequences in relation to health outcomes and/or interventions. This allows close study of clinical progression over different monitoring occasions but results in nested repeated measures (NRM) data that require more complex correlation structures [3, 4]. Meanwhile, several studies have found a strong association between obstructive sleep apnea (OSA) and cardiovascular morbidity and mortality [2, 5, 6]. Diagnosis and thus subsequent treatment of OSA, especially at young ages, are essential in decreasing cardiovascular morbidity and mortality and improving overall prognosis [5, 6].

Loss to follow-up or drop-out is a serious challenge in ABPM and other medical monitoring studies, yet the standard linear mixed-effects model for analysis of longitudinal measurements is often applied but does not account for such types of informative missingness. Joint modeling of the longitudinal marker of interest and the drop-out process includes a survival submodel to adjust the linear mixed-effects submodel. However, joint modeling has not been applied in NRM studies with nonlinear, heterogeneous outcomes like ABPM monitoring.

Joint models are widely used for analysis of longitudinal data with nonignorable drop-out. This method allows a model for the drop-out process to be fitted along with the usual longitudinal model of interest. Recently, a number of studies have provided alternative methods for handling informative missing data in longitudinal studies. Wu and Bailey [7] described a linear model for a continuous Gaussian distributed response using drop-out times as covariates in a random effects model. Other studies have focused on handling nonrandom drop-out in discrete longitudinal responses. Follmann and Wu [8] proposed a parametric generalized linear mixed model for binary data while adjusting for informative missingness. Similarly, Pulkstenis et al. [9] suggested a binary mixed-effects model for longitudinal ordinal responses with nonrandom drop-out. However, these models commonly use time-dependent covariate slopes, which do not directly take into account the structure of NRM data.

For these reasons, we propose an approach that utilizes advantages of joint modeling in the shared parameter framework. Our method includes linear mixed-effects regression with orthonormal splines to estimate nonlinear diastolic blood pressure (DBP) trajectories in the longitudinal submodel. This newly developed joint model offers flexibility in modeling NRM while still accounting for informative drop-out and providing an extension for the random effects structure beyond the established joint model framework. Not accounting for these features could bias estimates of the DBP trajectories. Another interesting feature of our application to the nested 24-hour ABPM data in the proposed joint model framework is the large number of repeated measurements, which is a relatively new phenomenon in clinical studies. Nevertheless, these collections of DBP sequences pose problems of multicollinearity due to correlated measurements. We therefore propose restricted cubic splines in a mixed-effects submodel as a novel application to alleviate this problem and allow for accurate modeling of DBP trajectories. Our objectives are to identify clinical covariates associated with DBP trajectories and/or drop-out propensity and to understand how those associations compare to those found with conventional modeling using the two-stage approach, wherein the longitudinal model is fitted first, and its empirical estimates are subsequently added when fitting the time-to-event model.

In Section 2, we introduce the motivating data with summary statistics on drop-out patterns. In Section 3, we describe the proposed joint model with extended random effects for NRM, together with implementation of this model, and we compare it to the currently available two-stage model. We apply the models in Section 4.  Section 5 details simulation study findings.  Section 6 concludes with remarks on our approach and application, along with future work.

## 2. ABPM Data and Missingness

Our approach was motivated by a prospective longitudinal study investigating the effects of surgical intervention on 24-hour ABPM in OSA. The study protocol outlined that DBP profiles were to be observed at half-hourly intervals beginning with the time of sleep onset for each subject. Details of this study have been described elsewhere, including application of conventional linear mixed-effects models [10, 11]. The original study recruited a total of 178 children consisting of individuals classified into one of three experimental groups based on overnight polysomnography: severe OSA, mild OSA, or healthy control. The goal was to evaluate the changes over time in DBP profiles from children with mild or severe OSA after surgical intervention (adenotonsillectomy), compared to profiles observed on healthy controls. The study consists of four separate periods, each with 24-hour blood pressure monitoring at 30-minute intervals: visit A (preintervention or baseline); visit B (1.5 months postintervention); visit C (6 months postintervention); and visit D (one-year postintervention). Control subjects were followed using the same visit schedule. A prior study of a novel clustering method utilized baseline data from this cohort but did not address repeated measures from follow-up visits [12].  Figure 1 exemplifies the visit-specific profiles of three subjects who completed the entire study duration, demonstrating the within-subject variability arising from the inner-repeated measure (within a given 24-hour interval) and the outer-repeated measure (visits A-D). Furthermore, within a given visit, there is heterogeneity between subjects and also within each subject over the 24-hour interval. An added complexity is that the circadian rhythm, which is inherent in the underlying longitudinal DBP process, is noisily measured. Baseline demographic/clinical characteristics of the subjects are summarized in Table 1.

A common challenge in longitudinal studies in the clinical setting is the occurrence of dropout while collecting long-term follow-up information for each subject [13–15].  Table 2 summarizes missing data patterns arising from drop-out from visits A to D. Nearly 67% of children have at least one missing DBP profile from visit B to visit D, while 33% had DBP observations for all visits. Inspecting patient characteristics can provide insights into the reasons for dropout [16]. The divergence in drop-out rates between treatment arms may be due to perceived benefits, in which case it is of considerable clinical significance to understand the drop-out mechanism [17].  Figure 2 provides the Kaplan-Meier curves of time to drop-out by group. All groups completed baseline (visit A). The probability of remaining in the study decreased at different rates between groups. Notably, the severe group had the highest rate of drop-out, which is interesting because this group is expected to require the most medical attention. Median drop-out time and 95% CI are reported in Table S1 in the supplement: study time to drop-out by group. Median drop-out times for control, mild, and severe groups were 365, 273, and 21 days, respectively. There was no significant difference between baseline characteristics of subjects who completed the study period from those who dropped out as described in Table S2: baseline characteristics of the study cohort by drop-out status. These results are in line with logistic regression analysis, which used drop-out status as the outcome variable as shown in Table S3: logistic regression model of drop-out status.

Although missing data mechanisms cannot formally be tested, exploratory analyses suggest that dropout is likely to be informative, given relevance to patient characteristics, in particular disease severity, and the observation that dropout occurred at differing rates between the groups. Given that the severe group dropped out at the highest rate (35%), it is possible that perceived treatment benefit from surgical intervention could have played a role in “sicker” subjects' willingness to discontinue the study.

## 3. Joint Modeling of ABPM Data

We present an overview of shared parameter models for informative dropout with discussion of missing data mechanisms in the context of the motivating data in Section S2 of the supplement. Reviews of missing data concepts and model frameworks have been provided elsewhere [13, 18–26]. For this study, we assume the data are missing not at random (MNAR) and use the shared parameter framework to develop a corresponding joint model for the outcome and missingness. Our approach links the longitudinal submodel and time to the dropout submodel by sharing a set of random effects for each individual. The main aim of our application is to identify patient characteristics that can potentially influence the DBP trajectories and informative dropout. We propose the methodology along the lines of Follmann and Wu [8], but we extend it for NRM data, which occurs often in the context of recurrent medical monitoring. This extension also enables greater utility for joint models in settings with intensely collected data.

### 3.1. Longitudinal DBP Submodel

A linear mixed-effects model with random intercepts and slopes is one of the most commonly used submodels for characterizing a longitudinal process measured through continuous data in a joint model [27, 28]. The random effects vector is extended to incorporate the NRM data structure as follows.

Consider the Gaussian linear-mixed-effects model for NRM data. Suppose there are *n* patients in the DBP study indexed by *i* = 1, 2, ⋯, *n*. Let DBP_*ijk*_ represent the DBP measurement for the *i*^th^ patient (*i* = 1, ⋯, *n*) taken at the *j*^th^ visit (*j* = 1, 2, 3, 4), at time *t*_*ijk*_(*k* = 1, ⋯, *n*_*ij*_) during the 24-hour interval. The measurements are recorded at time *t*_*ijk*_ which can vary between subjects, resulting in mistimed data. The *r*^th^ group (*r* = 1, 2, 3) corresponds to control, mild, and severe designation. We consider a general model for longitudinal DBP trajectories that account for the NRM structure as described in previous work involving a single (as opposed to joint) model [3, 4].

(1) $$\begin{array}{c} \log{\left(\text{DBP}\right)}_{ijk}=\mu_{i}\left(t_{ijk}\right)+\epsilon_{ijk}=X_{i}^{T}\left(t_{ijk}\right)\beta +f_{rj}\left(t_{ijk}\right)+Z_{i}^{T}\left(t_{ijk}\right)b_{i}+\epsilon_{ijk}, \end{array}$$

where the expected behavior of DBP at time *t*_*ijk*_, denoted as *μ*_*i*_(*t*_*ijk*_), is represented by *X*_*i*_^*T*^(*t*_*ijk*_) containing subject-level covariates (BMI and race as shown in Table S4 in Section S1: baseline characteristics of the study cohort by group) and parameter vector for fixed effects **β**. It is worth noting that our model allows for time-varying covariates, although our application utilizes covariates measured once at baseline. The term *f*_*rj*_(*t*_*ijk*_) refers to the functional form of the population-level DBP trajectory; *Z*_*i*_^*T*^(t_*ijk*_) refers to the subject-specific random effects design matrix. In our model, this is represented as follows:

(2) $$\begin{array}{c} Z_{i}^{T}\left(t_{ijk}\right)b_{i}=b_{0i}+b_{1ij}\text{Visi}{\text{t}}_{ij}+b_{2ik}t_{ijk}, \end{array}$$

where **b**_**i**_ = (*b*_0*i*_, *b*_1*ij*_, *b*_2*ik*_)^*T*^ is the random effects vector that follows a multivariate Gaussian density with mean 0 and variance-covariance matrix *D*. The term *b*_0*i*_ is the random intercept for the *i*^th^ subject and characterizes how the overall mean of the DBP response function varies between subjects; *b*_1*ij*_ is the random effect for the *i*^th^ subject at the *j*^th^ visit and characterizes how two DBP responses vary at the same time between two separate 24-hour visits; *b*_2*ik*_ is the random effect for the *i*^th^ subject at the *k*^th^ time point and characterizes how an individual's DBP measurements vary within a single 24-hour visit. Lastly, we assume measurement error *ϵ*_*ijk*_ ~ *𝒩*(0, *σ*_*ϵ*_^2^), **b**_**i**_⊥*ϵ*_*ijk*_ for all *i*, *j*, *k* from (1).

#### 3.1.1. Spline Fitting

Natural cubic splines provide a powerful method to model mean profiles with nonlinear trajectories as presented in (Figure 1) and discussed in other works [29, 30]. Multicollinearity is a substantial obstacle when it comes to the use of natural cubic splines in the analysis of ABPM studies, resulting in very large values of the basis matrix and convergence problems [31]. To overcome this issue, orthonormal polynomials are used to provide a more accurate and stable model. Orthonormal polynomials are normalized in confined intervals (−1,1). This use can result in fewer errors and better handling of very large (or small) regression coefficients [29, 31]. We use the Gram-Schmidt orthogonalization process to find an orthogonal basis from a nonorthogonal basis.

Transformed natural splines with *l* = 5 internal knots were chosen based on quantiles of time at distinct locations, as described in Ngo and Wand [32] which yield basis functions based on (2):

(3) $$\begin{array}{c} f_{rj}\left(t_{ijk}\right)=\overset{L}{\underset{l=1}{\sum }}\zeta_{l}B_{n}\left(t_{ijk},\lambda_{l}\right)+\overset{L}{\underset{l=1}{\sum }}\zeta_{\text{l}}B_{n}\left(t_{ijk},\lambda_{l}\right)*\text{Visi}{\text{t}}_{j}+\overset{L}{\underset{l=1}{\sum }}\zeta_{l}B_{n}\left(t_{ijk},\lambda_{l}\right)*\text{grou}{\text{p}}_{r}+\overset{L}{\underset{l=1}{\sum }}\zeta_{l}B_{n}\left(t_{ijk},\lambda_{l}\right)*\text{Visi}{\text{t}}_{j}*\text{grou}{\text{p}}_{r}. \end{array}$$

A sensitivity analysis was performed to select the number (*L*) and location of the knots (*k*_*l*_ for each *l*). Knots for the evolution of DBP were chosen a priori through fitting the longitudinal submodel separately using maximum likelihood and Akaike Information Criterion (AIC). The knot set with lowest AIC was chosen as the preferred model. Further sensitivity analysis was conducted to test the main effects of visit and group, and the interaction effect between visit and group as linear functions using a previously described approach in medical monitoring studies [33, 34]. This resulted in each group and visit combination being represented with distinct spline coefficients.

### 3.2. Dropout Submodel

Recently, it has been argued that leaving the baseline hazard unspecified can lead to an underestimation of standard errors of the parameter estimates in joint models [35, 36]. We employ a common choice for modeling the baseline hazard parametrically, using the Weibull hazard [37]. Let *T*_*i*_ denote the time to experience the event of interest, timing of study drop-out, for the *i*^th^ subject. In the event submodel, we assume that the survival time follows a Weibull distribution; that is, *t*_*i*_~ Weibull where *θ*_*i*_(*t*) = exp{**w**_**i**_^*T*^*γ* + *α*^*T*^**b**_**i**_} and *N* > 0 is the shape parameter. The hazard at time *t* for the *i*^th^ patient is given by the following equation.

(4) $$\begin{array}{c} h_{i}\left(t\right)=N\;t^{N-1}\exp\left\{w_{i}^{T}\gamma +\alpha^{T}b_{i}\right\}=N\;t^{N-1}\exp\left\{w_{i}^{T}\gamma +\alpha_{0}b_{0i}+\alpha_{1}b_{1i}+\alpha_{2}b_{2i}\right\}, \end{array}$$

which monotonically increases with time if *N* > 1, decreases if *N* < 1, and remains constant if *N* = 1 [14, 24, 38]. In our application, the vector **w**_**i**_ has elements in common with *X*_*i*_ in (1), and parameter vector **γ** represents the corresponding effects. We note that the elements may differ between the two submodels and typically depends on the data/study context. The vector **α** relates the DBP responses and the dropout via the set of random effects vector **b**_**i**_. The covariates in the Weibull submodel are represented by

(5) $$\begin{array}{c} w_{i}^{T}\gamma =\gamma_{0}+\gamma_{1}\text{ag}{\text{e}}_{i}+\gamma_{2}\text{white}.\text{rac}{\text{e}}_{i}+\gamma_{3}\text{male}.\text{gende}{\text{r}}_{i}+\gamma_{4}\text{BM}{\text{I}}_{i}+\gamma_{5}\text{mild}.\text{grou}{\text{p}}_{i}+\gamma_{6}\text{severe}.\text{grou}{\text{p}}_{i}. \end{array}$$

### 3.3. Comparison with Available Two-Stage Approach

#### 3.3.1. Two-Stage Analysis

Tsiatis et al. [28] proposed estimating the joint model through a two-stage model. In step one, the Gaussian linear mixed-effects model is used to fit the longitudinal DBP data without consideration of the informative missingness. In step two, the estimated individual random effects from the linear mixed-effects model are included as covariates in the Weibull time-dependent model:

(6) $$\begin{array}{c} h_{ijk}\left\{t\;|\;\theta_{ijk}\left(t\right)\right\}=Nt^{N-1}\exp\left\{w_{i}^{T}\gamma +\alpha_{0}{\hat{b}}_{0i}+\alpha_{1}{\hat{b}}_{1ij}+\alpha_{2}\;{\hat{b}}_{2ik}\right\}. \end{array}$$

The main advantage of this method is its computational simplicity. Further, it is easy to implement using existing software. However, a major drawback of using the two-stage approach is when there is informative dropout. In such cases, there is bias and loss of efficiency by not considering the time-to-event information when modeling the longitudinal process [23, 39]. Despite these drawbacks, it is the currently available approach if implementing joint models with an NRM structure.

### 3.4. Estimation and Sampling

We utilized a Bayesian approach to estimate the posterior distributions of the parameters of the joint model. We used vague proper prior distributions for all parameters. For the regression parameters in both submodels (**β**, **γ**) and for the association parameters **α**, we used a multivariate Gaussian prior with mean vector 0 and precision matrix 0.01**I**, where **I** is the identity matrix. For the measurement error variance *σ*^2^, we used an Inverse Gamma prior with a large-scale parameter. For the random effects covariance matrix *D*, we used a noninformative multivariate Inverse-Wishart distribution with degrees of freedom equal to 3 (the number of random effect components) [24, 40]. Finally, for the regression coefficients of the Gram-Schmidt transformed natural spline, we set a multivariate Gaussian prior with mean vector 0 and precision matrix 0.01**I**. We implemented the joint model by creating a Markov Chain Monte Carlo (MCMC) algorithm via the R2WinBUGS version 2.1-21 library in the statistical package RStudio version 1.0.136 [41, 42]. We used a single MCMC chain with starting values of the parameter estimates from the two-stage approach for 150,000 iterations after we discarded the first 100,000 iterations as the burn-in phase. In order to reduce autocorrelation between samples, the iterations were thinned by sorting every 10^th^ iteration. As a result, the posterior mean of the parameters is based on 5,000 iterations. The convergence of the chain was monitored through trace plots. The two-stage approach was easy to apply in the Frequentist framework since there are available packages using lme4 and survival libraries in R. The WinBUGS codes for the proposed method are available in Section S5 in the supplement.

## 4. Application to ABPM Study Data

Parameter estimates for the joint and two-stage models fit to the study data are shown in Table 3. Being white and having higher BMI at baseline were associated with an overall increase in DBP trajectory based on our joint model results. The hazard function estimated from the dropout submodel decreased over follow-up. Whites dropped out less frequently according to the joint model.

Findings from the two-stage model partially corroborate the joint model findings, but effect estimates differed. Association between white race and DBP was positive but had higher magnitude, while the positive association between baseline BMI and DBP had lower magnitude. The hazard function was estimated as not changing over follow-up. Between-subject variation was estimated to be lower, but the random coefficient estimate for slopes was higher. With regard to the association parameters, both the joint model and the two-stage approaches indicate that the log(DBP) trajectory is associated with risk of dropout. In the joint model, the random effects for intercept and visit (${\hat{\alpha }}_{0}$ and ${\hat{\alpha }}_{1}$) implied that higher start values along the log(DBP) trajectory correspond to a decreased hazard of drop-out: HR = exp(−2.78) = 0.062 for every one-unit increase in log(DBP); 95% CI: (0.005, 0.943).

An increase in the log(DBP) trajectory from one visit to the next visit corresponds to a decreased hazard of drop-out: HR = exp(−22.99) ≈ 0, i.e., negligible. However, among estimates from the two-stage approach, only the random slope estimate ${\hat{\alpha }}_{2}$ was statistically significant. This suggests that positive rates of change in the log(DBP) trajectory correspond to decreased but relatively negligible hazard of drop-out: HR = exp(−19.50) ≈ 0.

The population-level DBP trajectory of the control group was stable between visits (Figure 3), but we observed that two-stage estimates for group effect estimated higher DBP over the 24-hour interval. Differences between the joint and two-stage models over nighttime were slight, but the models diverged from wake (about 8 hours from the time since sleep onset) until the end of the interval. We observed this trend for all four visits. Similarly, differences over visits in the mild group between the two models were minimal for early hours but later diverged (Figure 4). From joint modeling, the severe group tended to have a sharp increase around wakefulness, followed by gradually increasing DBP through the daytime (Figure 5); this pattern was not detected in the two-stage model. The two-stage model fits a similar pattern for severe as for the mild and control groups.

To compare the adequacy of the joint model and two-stage approach, we examined three different criteria based on observed and estimated log(DBP) values: mean absolute error, root-mean-square error, and mean absolute percentage error (MAPE). The results show that the joint model and the two-stage approach both performed with excellent accuracy, e.g., MAPE for the joint and two-stage models were 2.3% and 2.0%, respectively. Table S5 in Section S3 of the supplement: model comparison results show that the joint model and the two-stage approach both performed with excellent accuracy, e.g., MAPE for the joint and two-stage models were 2.3% and 2.0%, respectively. Equations for these metrics are also provided in Section S3.

## 5. Simulation Studies

To assess the performance of the proposed joint model, we conducted simulation studies to mimic the study data that motivated this research. In the first step, a complete dataset including covariates as well as longitudinal responses across four visits was generated under a multivariate Gaussian distribution. In the second step, longitudinal responses were set to dropout timing via a Weibull hazard model. Due to the heavy computational load, we limited the number of simulations to *p* = 20. Each simulated dataset contained 200 individuals, and the MCMC algorithm ran with a single chain for 120,000 iterations, with a burn-in of 100,000 and thinning of 10.

### 5.1. Simulation of Complete Data

For each simulation, a complete longitudinal outcome *Y* was generated via the following model:

(7) $$\begin{array}{c} Y_{ijk}=\delta_{0}+\delta_{1}t_{ijk}+\delta_{2}\text{severe}.\text{grou}{\text{p}}_{i}+\delta_{3}\text{visit}.{\text{B}}_{ij}+\delta_{4}\text{visit}.{\text{C}}_{ij}+\delta_{5}\text{visit}.{\text{D}}_{ij}+b_{0i}+b_{1ij}\text{visi}{\text{t}}_{ij}+b_{2ik}t_{ijk}+\epsilon_{ijk}, \end{array}$$

where *y*_*ijk*_ corresponds to log(DBP) measurements for *i*^th^ subject taken at *j*^th^ visit and *k*^th^ time point. All terms are defined and distributed as in (1) except for simplicity, we assume *μ*_*i*_(*t*_*ijk*_) follows a linear trend at each visit and that there are only two experimental groups. Measurement error was generated using *σ*_*ε*_^2^ = 2.302, and variance-covariance terms for random effects **b**_**i**_ in (2) were generated as *σ*_*b*_0*i*__^2^ = 0.1, *σ*_*b*_0*i*_,*b*_1*ij*__ = 0.01, *σ*_*b*_0*i*_,*b*_1*ik*__ = 0.04, *σ*_*b*_1*i*__^2^ = 0.1, *σ*_*b*_1*ij*_,*b*_1*ik*__ = 0.02, and *σ*_*b*_1*ik*__^2^ = 0.1. Fixed-effects parameters were set to *δ*_0_ = 4.094, *δ*_1_ = 2.302, *δ*_2_ = 0.4054, *δ*_3_ = 0.6930, *δ*_4_ = 0.4050, and *δ*_5_ = −0.6930.

### 5.2. Generation of Missing Outcome

Once the complete dataset was generated, a nonignorable missing data mechanism was induced for log(DBP) through patient dropout where true time to dropout, *T*_*i*_, was generated assuming a Weibull distribution with hazard rate that depended on the covariates control group or severe group, and the set of random effects **b**_**i**_ as defined in (7):

(8) $$\begin{array}{c} h_{i}\left(t\right)=N\lambda {\left(t\right)}^{N-1}\exp\left\{\gamma_{1}+\gamma_{2}\text{severe}.\text{grou}{\text{p}}_{i}+\alpha_{0}b_{0i}+\alpha_{1}b_{1i}+\alpha_{2}b_{2i}\right\}. \end{array}$$

The shape parameter was set at *N* = 1 while the scale parameter was set at *λ* = 1. This yields approximately 30-40% dropout over a four-visit period. We set the parameter *γ*_1_ = 0.2; disease effect parameter was set as *γ*_2_ = 0.6931 with corresponding hazard ratios HR = 1.99 for diagnosis of severe OSA versus no OSA. For the association parameters, we considered *α*_0_ = −0.6931(HR = 0.50) corresponding to subjects with the same disease severity and lower log(DBP) at baseline being more likely to drop out; *α*_1_ = −0.9162 represents subjects with the same disease severity and increase in log(DBP) between visits corresponding to a decreased dropout hazard; *α*_2_ = −1.203 depicts patients with the same disease severity who exhibit a steeper decrease in longitudinal trajectory being more likely to drop out.

The observed follow-up times are given by *T*_*i*_^∗^ = min{*T*_*i*_, *C*} referring to the minimum of the true dropout and censoring times. We simulate *C* from an exponential distribution with a rate of 4. Finally, the event indicator equals one if the true dropout time is less than or equal to the censoring time. In order to induce missingness through visits, we used the following indicators:

(9) $$\begin{array}{c} \text{Event}=\left\{\begin{array}{cc} \text{dropped out at visit B}, & \min\leq T_{i}^{*}<Q1,\\ \text{dropped out at visit C}, & Q1\leq T_{i}^{*}<Q3,\\ \text{dropped out at visit D}, & Q3\leq T_{i}^{*}\leq \max, \end{array}\right. \end{array}$$

where min, *Q*1, *Q*3, and max are the minimum, first quartile, third quartile, and maximum values of observed follow-up times, respectively.

### 5.3. Evaluation Criteria

Let *δ* be the true values from Equations (7) and (8) to be estimated as the average of values obtained by fitting data over the *p* simulations. The accuracy of the posterior mean estimates was assessed using percent bias and coverage probability of each credible interval [43].

Trace plots from simulations implied no convergence issues. The results of the simulation study are summarized in Table 4. The longitudinal submodel is estimated more precisely compared to the survival submodel. The estimated *δ* terms achieved lower mean square error (MSE), less bias, and equivalently high coverage in the estimation compared to the terms estimated in the time-to-dropout submodel *γ*_1_, *γ*_2_ and *α*_0_, *α*_1_, *α*_2_. This could be attributable to the rate of dropout events and an insufficient number of repeated measurements for later visits. According to the coverage probability (CP), the results indicate that overall, our model performs adequately under simulated circumstances.

## 6. Discussion

We have developed a Bayesian joint model for nonlinear, heterogeneous NRM data to investigate the effects of informative drop-out. Using motivating data from an ABPM interventional study, we characterized longitudinal changes in DBP from children with mild and severe OSA after surgical intervention at visit A, and we compared it to DBP levels in healthy controls. We demonstrated how the presence of informative drop-out complicates the analysis, since the majority of patients with severe OSA dropped out and therefore observed longitudinal DBP profiles were limited. Thus, when analyzing such data, ignoring the drop-out process can lead to biased results. Our proposed joint model allows the incorporation of informative missingness in the analysis of motivating data and provides efficient inference of the treatment effects. We found discrepant estimation in daytime DBP evolution between the joint and two-stage models.

A particularly appealing feature of our approach is that it accounts for NRM data, which we achieved by extending the random effects vector to incorporate the nested structure. The longitudinal trajectory of DBP is expressed by a Gaussian linear mixed-effects model incorporating subject-specific random effects, and its association with the time to drop-out is assessed using both our joint model and the conventional two-stage approach. Natural cubic splines are frequently used to model nonlinear longitudinal trajectories and to compare groups and visits in ABPM studies. The application of such splines to our DBP study results in a highly correlated basis matrix, which can lead to convergence problems. To overcome this issue, our approach for longitudinal measurements included orthogonal transformation of the natural cubic splines. Number and location of knots were chosen before implementing the proposed joint model. Future work could focus on adaptive knot selection as part of the MCMC through methods such as reversible jump [44]. Potential differences between our chosen approach and use of penalized splines warrant further investigation.

Both the joint model and two-stage approach suggested effects of race, and BMI existed on DBP trajectories, as well as significant effects of race on the hazard of drop-out. Furthermore, the joint model indicated that patients who have a lower starting DBP are more likely to drop out. Our simulations indicated that the proposed model, particularly parameters from the drop-out submodel, may suffer from slight bias. Nonetheless, the application results suggest that additional insights may be gained through jointly modeling the informative drop-out using a simultaneous approach.

Limitations of the proposed joint model were mainly computational. In the application, the combination of sufficiently large sample size, high percentage of drop-out, high variability, and multiple visits led to challenges in the model estimation for some parameters. Higher rates of drop-out were investigated, including 50%, 60%, and 80%. All three rates resulted in the failure of the proposed joint model algorithm. These findings are directly in line with recent work [45]. Analysis of the ABPM data with a parametric Weibull submodel required approximately 28.16 hours to run for a single chain with 150,000 iterations. Our simulation study with moderate sample size still took about 2 hours for each replicate. The other limitation is that the proposed model may be influenced by prior distributions for unknown parameters. Our joint model for NRM data could be extended to a multivariate joint model to handle additional longitudinal outcomes [46–50]. For example, associations between systolic blood pressure and DBP processes could be assessed in conjunction with hypertension status and/or hazard of drop-out. Our joint modeling approach may be extended to include time-dependent covariates in both submodels, such as BMI which can vary over follow-up. The proposed model may be extended to explore different structures of association parameters, such as a shared parameter for area under the curve of the DBP trajectory, which may be associated with hazard of dropping out or onset of other medical conditions in ABPM studies. Extant studies are needed to assess the model's external validity.

## Figures and Tables

**Figure 1:** Three subject-specific profiles recorded during of 24-hour log (DBP) versus time since sleep onset (in hours) for four visits: visit A—baseline, visit B—1.5 months post-intervention, visit C—6 months post-intervention, and visit D—12 months post-intervention. Each subject's profile is marked between visits with a unique line color.

**Figure 2:** Plot of survival curves of drop-out in DBP data.

**Figure 3:** Control group's mean DBP evolution (log scale, *y* axis) over 24 hours (time since sleep onset, *x* axis) at each visit. Obtained from the two-stage (blue solid line), and the joint models (red solid line) with 95% CI (dashed line).

**Figure 4:** Mild group's mean DBP evolution (log scale, *y* axis) over 24 hours (time since sleep onset, *x* axis) at each visit. Obtained from the two-stage (blue solid line), and the joint models (red solid line) with 95% CI (dashed line).

**Figure 5:** Severe group's mean DBP evolution (log scale, *y* axis) over 24 hours (time since sleep onset, *x* axis) at each visit. Obtained from the two-stage (blue solid line), and the joint models (red solid line) with 95% CI (dashed line).

**Table 1:** Baseline characteristics of the pediatric participants (*N* = 178).

Characteristics^∗^	No. of children	Mean (SD) or %
Age at baseline (in years)	178	10.45 (2.21)
BMI at baseline (*z*-score)	178	0.85 (1.19)
Race (white)	178	61%
Gender (male)	178	48%
Experimental group		
Control	61	34%
Mild	61	34%
Severe	56	31%

BMI: body mass index; ^∗^Baseline defined as visit A; *z*-scores were computed according to Centers for Disease Control and Prevention growth charts.

**Table 2:** Dropout patterns of DBP trajectories (visits A-D).

Visits	Visit A	Visit B	Visit C	Visit D	Drop-out per pattern	%
No. observed	178	97	78	58		
	✓	✓	✓	✓	—	0%
	✓	✗	✗	✗	81	46%
	✓	✓	✗	✗	19	20%
	✓	✓	✓	✗	20	26%

DBP: diastolic blood pressure; ✓ = DBP is observed; ✗ = DBP is missing.

**Table 3:** Parameter estimates for DBP and informative dropout association based on the joint model and two-stage approach.

Parameter estimate	Joint model			Two-stage model^∧∧^		
Longitudinal submodel for DBP^∧^	Mean	SD	95% CI	Mean	SD	95% CI
White race (${\hat{\beta }}_{1}$)	2.9155	0.0919	(2.6600, 3.0470)^∗^	4.0091	0.0100	(3.9800, 4.0300)^∗^
BMI *z*-score (${\hat{\beta }}_{2}$)	0.7068	0.0067	(0.5653, 0.8165)^∗^	0.0086	0.0000	(0.000, 0.017)^∗^
Variation components, random effects						
Between subjects, intercepts $\left({\hat{\sigma }}_{b_{0}}^{2}\right)$	5.6011	0.6043	(4.5209, 6.8862)^∗^	0.0600		
Covariance, intercept, and visits $\left({\hat{\sigma }}_{b_{0},b_{1}}\right)$	−0.1881	0.0405	(−0.2781, −0.1170)^∗^			
Covariance, intercept, and slopes $\left({\hat{\sigma }}_{b_{0},b_{2}}\right)$	0.0112	0.0167	(−0.0214, 0.0439)			
Between subjects, visits $\left({\hat{\sigma }}_{b_{1}}^{2}\right)$	0.0246	0.0046	(0.0171,0 .0353)^∗^	0.0400		
Covariance, visits, and slopes $\left({\hat{\sigma }}_{b_{1},b_{2}}\right)$	−0.0006	0.0011	(−0.0027, 0.0014)			
Between subjects, slopes $\left({\hat{\sigma }}_{b_{2}}^{2}\right)$	0.0058	0.0006	(0.0047, 0.0071)^∗^	0.0400		
Measurement error $\left({\hat{\sigma }}_{\varepsilon }^{2}\right)$	0.0159	0.0002	(0.0156, 0.0162)^∗^	0.1200		
Weibull submodel for dropout						
Shape ($\hat{N}$)	0.7388	0.1035	(0.5456, 0.9610)^∗^	1.0000	1.0300	(0.9600, 1.0400)
Intercept (${\hat{\gamma }}_{0}$)	4.6567	5.2972	(−6.2182, 14.0500)			
Age (${\hat{\gamma }}_{1}$)	−0.0365	0.0609	(−0.1572, 0.0818)	−0.0000	0.03900	(−0.2900, 0.4400)
Male gender (${\hat{\gamma }}_{2}$)	−0.2594	0.2658	(−0.7776, 0.2553)	0.0680	0.1870	(0.0680, −0.2500)
BMI *z*-score (${\hat{\gamma }}_{3}$)	−1.7578	0.9144	(−3.3892, 0.1121)	0.0800	0.0800	(−0.7600, 0.2500)
White race (${\hat{\gamma }}_{4}$)	−8.2174	3.8876	(−15.5100, −0.2371)^∗^	−0.2400	0.1900	(−0.6200, 0.1300)
Mild group (${\hat{\gamma }}_{5}$)	−0.4286	0.3381	(−1.1130, 0.2078)	0.1500	0.2300	(−0.3000, 0.6000)
Severe group (${\hat{\gamma }}_{6}$)	−0.1986	0.3650	(−0.9393, 0.5088)	0.2400	0.2300	(−0.2200, 0.6900)
Random effects						
Random intercepts (${\hat{\alpha }}_{0}$)	−2.7811	1.3194	(−5.2860, −0.0579)^∗^	−1.4000	1.9700	(−5.2700, 2.4700)
Random visits (${\hat{\alpha }}_{1}$)	−22.9998	3.6157	(−30.3305, −16.1298)^∗^	−1.1700	3.2700	(−7.5700, 5.2300)
Random slopes (${\hat{\alpha }}_{2}$)	−1.3591	9.8496	(−20.4918, 18.0111)	−19.5000	4.3200	(−27.9700, −11.0200)^∗^

BMI: body mass index; CI: credible interval; DBP: diastolic blood pressure; SD: standard deviation of parameter estimate. ^∧^Group-specific splines included in the longitudinal submodel are reported in the supplement. Tables S6 and S7 in Section S4: the coefficients of the transformed natural cubic spline functions for the two-stage approach and the joint model; ^∧∧^parameter estimates evaluated using Wald test; ^∗^95% CI excludes 0.

**Table 4:** Simulation study results for the joint model with NRM.

Parameter	True value	Mean	Bias (%)
Longitudinal submodel for DBP			
Intercept (*δ*_0_)	4.0940	4.0912	−0.0758
Time (*δ*_1_)	2.3020	2.2933	−0.4019
Severe group (*δ*_2_)	0.4050	0.4167	2.7718
B visit (*δ*_3_)	0.6930	0.6872	−0.8514
C visit (*δ*_4_)	0.4050	0.4011	−1.0876
D visit (*δ*_5_)	−0.6930	−0.7019	1.2641
Weibull submodel for drop-out			
Intercept (*γ*_1_)	0.2000	0.2056	2.7844
Severe group (*γ*_2_)	0.6931	1.0621	53.2295
Random intercepts (*α*_0_)	−0.6931	−0.6583	−5.0249
Random visits (*α*_1_)	−0.9162	−1.2610	37.6157
Random slopes (*α*_2_)	−1.2030	−1.5865	31.7724

Parameter	SE	MSE	CP (%)

Longitudinal submodel for DBP			
Intercept (*δ*_0_)	1.3646	0.8692	100
Time (*δ*_1_)	0.7943	0.1009	80
Severe group (*δ*_2_)	1.5891	1.5981	100
B visit (*δ*_3_)	1.1000	0.3664	100
C visit (*δ*_4_)	1.3868	0.9282	95
D visit (*δ*_5_)	1.6593	1.9051	95
Weibull submodel for drop-out			
Intercept (*γ*_1_)	3.3569	45.0296	100
Severe group (*γ*_2_)	3.8810	106.3326	90
Random intercepts (*α*_0_)	8.2471	2094.8071	95
Random visits (*α*_1_)	6.7220	1032.5449	90
Random slopes (*α*_2_)	5.5531	414.4210	100

CP: coverage probability; DBP: diastolic blood pressure; SE: standard error; MSE: mean square error.

## Data Availability

Data access has been restricted due to the sensitive nature of its contents. Anyone wishing to use the data may contact and request permission from the primary investigator of the original study (author RSA).

## Supplementary Materials

Supplementary Materials Implementation code, additional descriptive statistics of the study data, and results from model applications are available online.
